# ARIMA Model and Few-Shot Learning for Vehicle Speed Time Series Analysis and Prediction

**DOI:** 10.1155/2022/2526821

**Published:** 2022-01-19

**Authors:** Yingzi Wang, Ce Yu, Jue Hou, Sisi Chu, Yongjia Zhang, Yue Zhu

**Affiliations:** ^1^College of Intelligence and Computing, Tianjin University, Tianjin 300300, China; ^2^Automotive Data of China (Tianjin) Co., Ltd., Tianjin 300300, China

## Abstract

In the fields of traffic management, traffic health, and vehicle safety, vehicle speed prediction is an important research topic. The greater the difference between vehicle speed and average vehicle speed, or the more discrete the vehicle speed distribution, the higher the accident rate. This paper proposes a vehicle speed prediction method based on adaptive KF (Kalman filtering) in the ARMA (Autoregressive Moving Average) environment to address the problem of high-speed moving vehicle speed prediction. The ARMA theory is used to model the prediction of speed time series. The contribution rate of each coefficient representing the original time series is different after fitting the original time series with the ARMA model, so each coefficient must be given a certain weight. Multisource traffic data fusion and interval speed prediction are carried out on the basis of few-shot data preprocessing and traffic state division, according to different traffic states. The speed prediction accuracy is very high, according to the algorithm verification results.

## 1. Introduction

According to statistics, intersections account for roughly 30% of all traffic accidents [1]. Even when traffic control lights are installed at intersections, deadly collisions caused by illegal activities such as speeding and running red lights still occur. At intersections, drivers must pay attention to influencing factors such as vehicles traveling in different directions, pedestrians, and nonmotor vehicles, as well as the relative positions of their own vehicles, and then make driving behavior decisions in a short amount of time [2, 3]. If the driver can be given some information about his own vehicle's operation ahead of time, it will greatly reduce the driver's driving difficulty at the intersection.

When driving on the road, drivers set their own speed based on the terrain and road conditions [4]. When the road's horizontal, vertical, and horizontal geometric elements exceed the minimum requirements for safe driving of automobiles on this grade of road, and external conditions such as traffic density, terrain, and climate are favorable, the actual driving speed of automobiles often approaches or exceeds the design speed [5, 6]. Entering the intersection and arranging them according to the time mark, according to existing research, can not only reflect the characteristics of drivers' individual driving behavior. Time series differ from ordinary series in that the data are organized in chronological order, and each numerical point has a corresponding time point [7]. These data are generated as part of the day-to-day operations of businesses, hospitals, schools, and other institutions, and they gradually accumulate into a large-scale time series database. The two types of data can be mutually supplemented and verified using data fusion. The accuracy of vehicle speed prediction across corresponding regions will be improved as well.

The above-mentioned contents are the focus of this paper. ARMA (Autoregressive Moving Average) predictive modeling was used [8]. The time series of vehicle speed generated when the object to be evaluated (own vehicle) and the vehicle in the direction of conflict (other vehicle) drive to the intersection at the same time serves as the evaluation basis and modeling data. The modeling data come from a real-world vehicle driving test. Multisource traffic data fusion and interval speed prediction are carried out according to different traffic states using data preprocessing and traffic state division.

## 2. Related Work

The purpose of travel time prediction is to use historical and real-time distance, speed, traffic flow, travel time, or some variables mathematically related to travel time to obtain the travel time of vehicles that will leave at a certain time in the future and whose starting and ending points are determined [9, 10]. These known variables can be obtained through equipment collection, estimation, or prediction [11]. In the process of predicting the travel time of expressway, combining the travel time of different sections in different time periods, the traffic operation conditions of different sections are obtained, and the results are extended to the whole section of expressway, and the final travel time prediction result is obtained, with a good result of about 10% error%. Literature [12] studies the daily travel time model and applies linear regression and tree model to travel time prediction. The input parameters include traffic flow information, occupancy data collected by single-loop detector, and historical travel time information (Literature [13]). Using the data collected by point traffic detectors, a short-term expressway travel time prediction method is mined. They took into account the spatial and temporal changes of traffic data and made use of the traffic measurement data collected from different places at the current moment and different places at the historical moment to do this [14]. Using the ARIMA model to determine the potential hot spots of taxis, in the process of research, they regard the demand of passengers for taxis as a simple linearly changing structure, so only linear models are used to predict. Literature [15] puts forward a model for forecasting service demand, which is suitable for a single taxi station. The use of traffic flow data in the forecasting process is a comprehensive place for them to consider, and the model can be used for real-time forecasting in online environment. However, according to their research ideas, different taxi stations in the same city must carry out different model training in order to achieve more accurate prediction results.

The speed information of vehicles before entering the intersection can be used as the basis of vehicle collision risk assessment at the intersection. Literature [16] studies the probability model between the speed of vehicles heading for the intersection and the occurrence of collision accidents, and there is a clear correlation between the speed and the acceptable gap in the workshop. Literature [17] puts forward a dynamic model and a communication model between vehicles after analyzing the characteristics and process of traffic conflicts at signalless intersections and sorts out a set of algorithms. Finally, the effectiveness of the algorithm is verified by computer programming simulation. Literature [18] developed a speed control device for vehicle turning left at intersection. Finally, the simulation results show that the device can really improve the safety of vehicle turning left at intersection. Literature [19] puts forward two strategies of setting left-turn phase and left-turn waiting area at intersections to improve the traffic quality at intersections. Literature [20] found that the intersection conflict simulated by software or model is very suitable for the actual intersection conflict research. Literature [21] holds that the occurrence of traffic accidents is mainly caused by the driver's mistakes, and the driver carries out a series of driving actions for a certain purpose, but the original driving intention cannot be realized due to the operation mistakes. Literature [22] establishes a hidden Markov model based on the pedal opening of the vehicle and the position information of the vehicle, so as to determine the intention that the driver really wants to achieve. Reference [23] establishes a hidden Markov model to infer the driver's intention when the vehicle deviates to different degrees. The final reasoning result is applied to the control device of the vehicle, which increases the safety of the vehicle when driving.

In order to determine the driver's driving intention, all types of state data must be collected, and an identification model must be established during the analysis of the driver's driving. The challenge is deciding what kind of data to collect, or choosing the feature vector for modeling. The difficulty of model building and the time it takes to identify a model can be reduced if the feature vector dimension is too small. However, the model's accuracy will deteriorate. Furthermore, collecting characteristic data in the actual driving environment of some vehicles is quite difficult. As a result, selecting the appropriate feature vector is critical in the study of predicting a driver's driving intention.

## 3. Research Method

### 3.1. Vehicle Speed Time Series Analysis

It is a critical variable in the field of speed traffic, and vehicle driving speed is a key index for reflecting traffic operations, and the driving state of floating vehicles can best reflect traffic operations over time. The traffic situation is constantly changing in real time, and the travel time of vehicles is directly influenced by the current traffic situation. As a result, understanding how to convert and correlate vehicle and traffic driving conditions, as well as how to display the short-term operation of traffic using appropriate variables, is critical. Under such conditions, road speed is generated.

In the research, this model is mainly used to calculate the traffic conditions before vehicles enter the expressway. When it is necessary to predict the travel time, the estimated travel time, the estimated starting point, and the expected ending point of the vehicle are all known. After getting the speed of the road section before the estimated travel time, then can know the traffic conditions during this period. At the same time, from the second 5 minutes to the first 5 minutes before the trip, one can get a general understanding of the changes in traffic operation. For the known estimated travel time, calculate the speed of each road segment within the first two 5 minutes of the trip, and arrange the speed of each road section according to the front and back position of the road section, so as to obtain the preliminary input characteristics.

In practical application, the complexity and unstructured degree of time series are very high, which forces the research to continuously improve the accuracy and applicability of time series mining algorithm. In reality, time series exists in all aspects. Finding the hidden rules and patterns from these complex data and finally serving for decision-making is the main purpose of data mining.

In the past research, the ARMA model was mostly used in forecasting. This paper mainly uses the ARMA model to extract features of time series. Determining the time series {*X*_*t*_,  *t*=1,2,…, *n*} can fit the ARMA model. We can find the basic model type judgment diagram in Figure 1.

If the accurate optimal value of (*p*, *q*) cannot be obtained by using autocorrelation function and partial autocorrelation function, AIC (Akaike information criterion) can be used to determine the order, which is a standard to measure the fitting effect of the model.

Increasing the parameter variables of the model will reduce the deviation between the estimated value of the model and the actual value, so that the model can better fit the original data. However, increasing the number of parameter variables will increase the complexity of the model, so the cost of increasing the variables should be punished.

The fitting ARMA model can be defined as follows:

(1) $$\begin{array}{c} \text{AIC}=\left(p,q\right)=N\;\ln\;\sigma^{2}\left(p,q\right)+2\left(p,q\right), \end{array}$$

where *N* is the sample size, *k*=*p*+*q* is the number of parameters in the ARMA model, and *σ*^2^ is the estimation of noise variance.

BIC (Bayesian information criterion) is also a judgment criterion, which is expressed as follows:

(2) $$\begin{array}{c} \text{BIC}\left(p,q\right)=N\;\ln\;\sigma^{2}\left(p,q\right)+\left(p,q\right)\ln\;N. \end{array}$$

The principle of this method is the same as that of AIC, but it increases the intensity of “punishment.” It can be seen that both of these criteria advocate the concise form of functions and use fewer variables to represent functions. When the number of samples is large, BIC principle is more effective, and AIC principle determines relatively many model parameters, so it is more suitable for small samples.

Check the autocorrelation and partial correlation between scattered data in time series data *X*_*t*_. By observing the distribution of autocorrelation and partial correlation function values, if the distribution curve accords with the characteristics of “tailing” and “truncated,” it shows that the series is suitable for establishing the ARMA model. The calculation formulas of autocorrelation *R*_*k*_ and partial correlation function *ϕ*_*k*,*k*_ for correlation judgment are as follows:

(3) $$\begin{array}{c} \left\{\begin{array}{c} R_{k}=E\left[X_{t},X_{t-k}\right],\\ \phi_{k,k}=\frac{E\left[X_{t},X_{t-k}\right]}{\sqrt{E{\left[X_{t}\right]}^{2},E{\left[X_{t-1}\right]}^{2}}},\;k=1,2,\ldots ,n. \end{array}\right) \end{array}$$

If the time series data do not meet the correlation requirements, it is necessary to perform differential, differential, or logarithmic operations on the data used for partial scatter points in *X*_*t*_ and then continue the subsequent steps when it becomes a stationary data series.

Select the appropriate *p*, *q* value to establish the analytical formula of ARMA model, and use the AIC rank criterion to determine the *p*, *q* value, even if the following formula is the minimum value:

(4) $$\begin{array}{c} \text{AIC}=\min\left[N\cdot \;\ln\;\delta_{k}^{2}+2\left(p+q+1\right)\right], \end{array}$$

where *N* is the capacity of the selected speed sample and *δ*_*k*_^2^ is the residual variance of the model, that is,

(5) $$\begin{array}{c} \delta_{k}^{2}=\sum_{k=1}^{N}\frac{\varepsilon_{k}^{2}}{N}. \end{array}$$

If the absolute values of residual autocorrelation functions of the prediction results are less than $2/\sqrt{N}$, it indicates that the ARMA model meets the prediction requirements.

In general, data can be divided into numerical and non-numerical types of characteristic attributes. These two types of filling are treated differently by the mean filling method. The missing values for numeric attributes will be filled using the average values of the attributes in other nonmissing samples. Fill in the values with the most frequent occurrences in the nonmissing samples, that is, the values with the highest frequency, for non-numeric attributes, according to the mode principle.

From the entire sample set, choose the road section speed that corresponds to the recorded road section and save it as the new adjacent road section sample set. Then, using a hierarchical clustering algorithm, this portion of the data is clustered, the centroid of each cluster is calculated, and the cluster centroid that is closest to the speed of the road section near the missing position is found. The values of data samples in the missing positions in the cluster are filled in the missing fields. This completes the missing item's filling.

### 3.2. Vehicle Speed Prediction

At present, the prediction method generally uses the previous historical data, taking the day as the cycle, extracting the change rule of traffic parameters from it, and applying the extracted rule to the current time, thus obtaining the prediction result. According to the comprehensive evaluation of the previous traffic state dividing thresholds, the specific dividing standards are determined.

After dividing the continuous traffic data into traffic states, the traffic data belonging to different traffic states are classified. According to the historical traffic data of each traffic state, the state transition matrix required by the KF (Kalman filtering) method is trained by the artificial neural network, and then the interval speed prediction based on data fusion is carried out by the KF method.

In the ARMA environment, the dynamic performance of high-speed moving vehicles is very high. Therefore, when the parameters change little, we use a larger adaptive forgetting factor *μ*_*k*_ to increase the prediction strength. When the parameters change greatly, a small adaptive forgetting factor *μ*_*k*_ is used to enhance the identification accuracy. The formula of adaptive forgetting factor used in this paper is as follows:

(6) $$\begin{array}{c} \mu_{k}=\max\left\{1,\frac{tr\left(G_{k}\right)}{tr\left(H_{k}\right)}\right\}. \end{array}$$

The core idea of memory decay is to apply a factor to the covariance matrix of prediction and increase the variance of prediction state vector, so as to make full use of the current measurement data.

(7) $$\begin{array}{c} G_{k}=M_{k}-{\text{CQC}}^{T}-R. \end{array}$$

In equation (7), *G*_*k*_ and *M*_*k*_ represents the error variance at time *k*.

(8) $$\begin{array}{c} H_{k}={\text{CAP}}_{k-1}A^{T}C^{T}. \end{array}$$

In equation (8), *H*_*k*_ represents the error variance at time *k*, which ensures that the value of the error covariance matrix *P*_*k*_ is symmetric and positive, and improves the dynamic performance of the system.

In this paper, the flow of speed prediction operation of high-speed moving vehicles based on adaptive KF in ARMA environment is shown in Figure 2.

The contribution weight also plays a role in reducing dimension and simplifying operation to a certain extent. On this basis, this paper puts forward a new similarity measurement standard, and the process of clustering analysis becomes the following steps.

Using the ARMA model to fit the model, the time series will be represented by a set of coefficient vectors. Namely, the time series *X*, *Y*, and the parameter vectors of the fitting model are *π*_*X*_, *π*_*Y*_, respectively.

Find the contribution rate (*α*_1_, *α*_2_,…, *α*_*m*_) of the first *m* coefficients whose cumulative contribution rate reaches a certain percentage and then calculate the weight *β*=(*β*_1_, *β*_2_,…, *β*_*m*_) of these *m* coefficients, where *β* is the weight vector and *i* represents the *i* th coefficient:

(9) $$\begin{array}{c} \beta_{i}=\frac{\alpha_{i}}{\sum_{i=1}^{m}\alpha_{i}}. \end{array}$$

The newly obtained coefficient vectors are standardized, their Euclidean distance *d*_*μ*_ is used as similarity measure, and the corresponding clustering method is used to recluster, and finally the clustering result is obtained.

(10) $$\begin{array}{c} d_{\mu }=\sqrt{\sum_{k=1}^{m}{\left(\mu_{Xk}-\mu_{Yk}\right)}^{2}}. \end{array}$$

Due to the weekly similarity of traffic data, historical data with the same weather conditions in the same week as the forecast date in the last week were selected in the study. If the weather conditions are different, select the data of the same week last week. If the weather conditions are still different, select the data of the adjacent Sunday of last week.

Because the one-dimensional median filter is less affected by the contour of image samples, and the noise suppression effect of the two-dimensional median filter is obviously better than that of the one-dimensional median filter when the contour of image is not considered, one-dimensional and two-dimensional median filters can be used alternately when filtering. In addition, during filtering, the image can be iteratively filtered to get the optimal solution.

## 4. Results Analysis and Discussion

### 4.1. Modeling and Analysis of Time Series Prediction

Design the real vehicle driving data collection test according to the vehicle collision situation. The driving area is selected at the intersection of a newly built municipal road, and it is required that the road connecting the intersection should extend long enough, have a wide field of vision, and have small traffic flow. Motor vehicles 1 and 2 in the direction of conflict use the same type of small cars, and the vehicle speed is collected once every 1 s by the vehicle driving behavior test platform and stored in chronological order.

After the vehicle stops, determine the position of the collision point according to the traveling direction of the vehicle and measure the distance from the starting point to the collision point, as shown in Figure 3.

In straight-line sections, drivers will first choose between three types of traffic crossing options based on their destination and intersection design: straight, left, or right. The external information, such as traffic lights/signs, other vehicles, pedestrians, nonmotor vehicles, roads and obstacles at intersections, weather factors, and so on, is primarily received visually. The driver will adjust his speed to prepare for entering the intersection based on the above factors. The driver primarily uses the accelerator and brake pedals to adjust the speed of his own car on the straight road section.

The driving in the straight-line section and the driving in the intersection follow each other on the time axis. The purpose of driving on the straight road section is to prepare for driving in the intersection, so the speed fluctuation on the straight road section reflects the driver's turning preparations.

If you go straight through the intersection, the driver's main gaze targets are the vehicles and traffic lights ahead. Compared with the other two turning modes of crossing, the influencing factors of straight-through crossing are relatively simple. However, the change of traffic lights directly affects whether the vehicle stops or not. Therefore, the speed of straight-through traffic varies greatly.

Comparing the degree of difference between the curves in Figures 4 and 5, it can be seen that the prediction model [20] established by using the first 40 data in the vehicle speed series obtained from the experiment has a better prediction effect on the last 20 vehicle speeds.

The vehicles run continuously in space, and the number and types of vehicles passing through different sections of each test section are basically the same in the same time period. However, for different observation points on the same section, the composition structure of vehicle types has spatial differences. In the process of driving on the expressway, certain drivers will frequently change lanes in order to choose the best route. This reflects the change of running speed in the direction.

By studying the speed change of different drivers when driving vehicles through the combination of curve and slope of the test section, the main influencing factors of drivers' driving behavior in the curve are found, so as to prepare for the later study of the running speed distribution characteristics of typical sections.

### 4.2. Verification and Analysis of Prediction Results

The vehicle will be acted on by centrifugal force pointing to the outside of the horizontal curve while driving on a curve. To improve the vehicle's lateral controllability, the driver typically slows down when entering the curve. The longitudinal stability of the vehicle is also involved in curve driving because the vehicle will decelerate when decelerating and the longitudinal stress will change. The safety of the entire route is largely determined by the quality of the curve's design, and curve speed characteristics have always been the focus of running speed research.

Because of the complexity and diversity of highway alignment composition, there are some differences in the running speed of entering the slope section, which affects the running speed of different sections on the slope section. Set at the longitudinal slope's beginning, middle, and end points, and increase the position section of the minimum sight distance point in the vertical curve section. You can track the vehicle to record the speed if the slope length is less than 800 meters. One person stands at the bottom of the slope or at the top of the slope, measuring the speed with a speed gun. Follow two people and keep track of their speed in two different directions. Because the speed measuring range of a radar speed measuring gun is limited when the slope is longer than 800 meters, more speed measuring personnel should be equipped. Record the relevant alignment and road surface parameters, roadside conditions, and road surface conditions of the point after the speed measurement test is completed, and take photos.

In the simulation experiment, three methods are used to predict the speed of high-speed vehicles. The predicted results of simulated vehicle speed are shown in Figures 6–8.

It can be seen from Figure 8 that during the whole iteration process, the maximum error between the actual running speed of the high-speed moving vehicle and the estimated speed based on the least square method is ±4 and fluctuates up and down here.

The original data obtained from the test include mileage, speed, and acceleration, which are continuously changing with the mileage. This paper mainly studies the distribution of running speed on curved slope sections, which are divided strictly according to the pile number. Therefore, the data obtained from the test should first be recalibrated according to the station number, so as to approximately get the continuous running state of vehicles on different sections.

The test shows that the mileage measured by the instrument is shorter than the actual pile number mileage. This is because the road pile number is based on the actual distance of the road centerline, and the instrument measures the actual mileage of the vehicle. However, when driving the vehicle, it is impossible for the driver to drive in strict accordance with the direction of the road centerline marking. Skilled drivers will often change lanes and choose shorter routes.

This kind of error caused by the driver's route selection is objective and inevitable in the test process, but the data can be recalibrated by setting special marking points, which are hereinafter referred to as “reference points.” Data calibration is actually an artificial dispersion of experimental errors, and the influence of this error can be reduced by increasing the number of “reference points” (Figures 9 and 10).

It can be seen from Figure 9 that the change trend of the predicted value is basically consistent with that of the real value. It can be seen from Figure 10 that the maximum relative error is 7.4, the error between the predicted result and the true value is small, and the predicted result is relatively accurate.

If you want to turn left through the intersection, the factors affecting the speed are more complicated than when you go straight through. Drivers should not only pay attention to the changes of traffic in intersections but also pay attention to the flow of people and nonmotor vehicles on crosswalks. According to the traffic rules, even if the traffic lights indicate that you can turn left, there are pedestrians and nonmotor vehicles crossing the street at the crosswalk.

The essence of the running speed method is to ensure the smooth and continuous running speed by controlling the gradual transition of the unit index values of adjacent road sections, thus improving the driving safety of the highway. In practice, the designer checks the consistency and coordination of technical indicators along the route direction through the running speed curve. If the vehicle speed curve under a certain set traffic volume is calculated, not only can you get the travel time between the start point and the end point, provide reference for road users' travel, but also measure the service level of the road, and then judge whether the design expectation is met and whether it is necessary to rebuild, expand, or build parallel lines.

## 5. Conclusion

This method improves KF's tracking ability by allowing it to record and predict the speed of high-speed moving vehicles in harsh environments, curves, uphill, and downhill. The predicted vehicle speed value is used to calculate vehicle displacement and distance between vehicles, which can be used to assess the risk of collisions in intersections between vehicles traveling in opposing directions. The research object is an ARMA model with a zero-mean random sequence. The simulation results show that the adaptive KF vehicle speed prediction method based on ARMA predicts values that are closer to reality, which improves the filter's convergence effect and reduces the fluctuation range, effectively overcomes the negative effects of process and measurement errors, and better reflects real-time effectiveness.

The vehicle speed prediction modeling and parameter tuning are done off-line, which is a flaw in this study. The ARMA modeling parameter self-tuning method and its implementation algorithm should be considered to help the prediction model adaptively adjust parameters to cope with changes in the driving environment, in order to improve the model's universality. The work described above will be continued in the follow-up study.

## Figures and Tables

**Figure 1:** Basic model type judgment. ACF is autocorrelation function, PACF is partial autocorrelation function, MA is the moving average model, and AR is the autoregressive model.

**Figure 2:** Adaptive KF speed prediction flow chart.

**Figure 3:** Time series of vehicle speeds 1 and 2 obtained from the real vehicle driving test.

**Figure 4:** Comparison between predicted value and measured value of vehicle 1.

**Figure 5:** Comparison between vehicle 2 predicted value and measured value.

**Figure 6:** Speed prediction effect of the least square method.

**Figure 7:** Speed prediction effect of KF.

**Figure 8:** Speed prediction effect of adaptive KF.

**Figure 9:** Comparison chart of data verification results.

**Figure 10:** Relative error diagram of data.

## Data Availability

The data used to support the findings of this study are available from the corresponding author upon request.
